The article "Manual Acupuncture at ST37 Modulates TRPV1 in Rats with Acute Visceral Hyperalgesia via Phosphatidylinositol 3-Kinase/Akt Pathway" was published in 2021. Journal: Evid Based Complement Alternat Med.

# Manual Acupuncture at ST37 Modulates TRPV1 in Rats with Acute Visceral Hyperalgesia via Phosphatidylinositol 3-Kinase/Akt Pathway

**DOI:** 10.1155/2021/5561999

**Published:** 2021-10-04

**Authors:** Caiyi Chen, Zhi Yu, Dong Lin, Xuan Wang, Xuejun Zhang, Feng Ji, Lingling He, Bin Xu

**Affiliations:** ^1^Key Laboratory of Acupuncture and Medicine Research of Ministry of Education, Nanjing University of Chinese Medicine, Nanjing 210029, China; ^2^School of Acupuncture and Moxibustion, Fujian University of Traditional Chinese Medicine, Fuzhou 350122, China

## Abstract

Acupuncture can significantly ameliorate inflammatory pain in acute visceral hyperalgesia. Hyperalgesia is attenuated by inflammatory mediators that activate transient receptor potential vanilloid 1 (TRPV1), and TRPV1 is regulated by nerve growth factor (NGF)-induced phosphatidylinositol 3-kinase (PI3K)/Akt pathway. However, it is unknown whether NGF-induced PI3K/Akt pathway is associated with manual acupuncture (MA). In this study, the effect and mechanism of MA at Shangjuxu (ST37) and Quchi (LI11) were examined using an acetic acid-induced rat model with visceral hyperalgesia. We demonstrated that MA at ST37 significantly decreased abdominal withdrawal reflex (AWR) scores, proinflammatory cytokine expression (TNF-*α*, IL-1*β*, and IL-6), and TRPV1 protein and mRNA expression in rats with acute visceral hyperalgesia compared with the untreated controls, while MA at LI11 showed no effect. The effects of MA at ST37 were reversed after treatment with the PI3K agonist IGF-1 30 min before MA. In rats with visceral hyperalgesia, the upregulation of NGF, tropomyosin-receptor-kinase A (TrkA), PI3K, and phosphorylation-Akt (p-Akt) was decreased by MA at ST37, indicating that TRPV1 regulation via the NGF-induced PI3K/Akt pathway plays a vital role in the effects of MA-mediated amelioration of acute visceral hyperalgesia.

## 1. Introduction

Visceral pain is a common type of pain caused by underlying disease, for which patients frequently seek medical intervention. According to the World Health Organization, 22% of primary care patients experience persistent pain [1], and about 11% of patients worldwide with abdominal pain have irritable bowel syndrome (IBS) [2]. The most common drugs currently used to treat acute and chronic visceral pain disorders include analgesics, antispasmodics, and antidepressants. However, these are frequently associated with adverse effects such as addiction and constipation [3].

Acupuncture, a traditional Chinese treatment, has been used in the clinic to improve visceral functions [4] and ameliorate acute [5–7] and chronic [8–11] pain. ST37 and LI11 are two the most effective acupoints for treating intestinal diseases [12–18]; however, they showed different analgesic effects in the model of zymosan-induced colorectal hypersensitivity [19]. Previous research studies found that the treatment effect of ST37 on the ulcerative colitis is better than LI11 in improving the ulcer score, whose mechanism is underlying alleviation of tumor necrosis factor (TNF)-*α* and increasing the levels of choline acetyltransferase (ChAT) and alpha 7 nicotinic acetylcholine receptor (*α*7nAChR) [20].

The proinflammatory cytokine like TNF-*α* could activate the peripheral receptors TRPV1 in pain transmission [21]. Hyperalgesia is induced by inflammatory and postinflammatory mediators that activate TRPV1, suggesting that TRPV1 plays a role in inflammatory pain [22, 23]. Recently, many studies have explored the efficacy of EA for the treatment of abnormal pain in chronic visceral hypersensitivity [24, 25] and acute visceral hyperalgesia [7, 26]. The efficiency of EA is thought to be correlated with the regulation of TRPV1 [10, 27]. NGF can bind the TrkA receptor and activate PI3K and Src kinase to phosphorylate TRPV1 [28]. However, the mechanisms underlying the effects of acupuncture are still unclear. In this study, we aimed to determine whether the effect of MA at LI11 and ST37 is different, and the regulation of TRPV1 expression by NGF-induced PI3K/Akt is involved in the mechanism of MA, using an acetic acid-induced rat model visceral hyperalgesia.

## 2. Materials and Methods

### 2.1. Animals

With reference to the study by Qi et al. [26], 36 male Sprague Dawley rats weighing 300–380 g were obtained from the Institutional Animal Care and Use Committee of Fujian University of Traditional Chinese Medicine (license number, SYXK [Fujian] 2014-0005). All rats were provided *ad libitum* access to water and food and were housed in specific pathogen free (SPF) facility under a 12 h light/dark cycle and standard conditions at 23°C ± 2°C. All experimental procedures were conducted in accordance with the NIH Guide for the Care and Use of Laboratory Animals.

### 2.2. Instrumentation

The ABI StepOnePlus RT-PCR instrument was purchased from Applied Biosystems (Foster, CA, USA), High Speed Refrigerated Centrifuge was obtained from Eppendorf (Hamburg, Germany), and Chemiluminescence Imaging Analysis System, Electrophoresis System, Trans-Blot Turbo Transfer System, and Microplate Absorbance Systems were purchased from Bio-Rad (Hercules, CA, USA).

### 2.3. Reagents

The PI3K agonist IGF-1 was purchased from Biovision (Milpitas, CA, USA), and a 0.1 mg/ml stock was prepared in saline. Tumor necrosis factor (TNF)-*α*, interleukin (IL)-1*β*, and interleukin (IL)-6 rat ELISA kits were obtained from Nanjing Jiancheng Bioengineering Institute (Nanjing, China). NGF, TrkA, PI3K, TPRV1, and *β*-actin antibodies were purchased from Abcam (Cambridge, UK). Akt, p-Akt (Ser473) antibodies, and secondary antibodies goat anti-mouse IgG were obtained from Proteintech (Rosemont, IL, USA). The secondary antibodies goat anti-rabbit IgG was purchased from Huabio (Hangzhou, China).

### 2.4. Modeling Procedure and Grouping

Acute visceral hyperalgesia was induced as reported by Qi et al. [26]. 36 rats were randomly allocated into the following groups with 6 in each group: (1) normal, (2) model, (3) ST37, (4) LI11, (5) ST37 + IGF-1, and (6) IGF-1. 1.5 ml of saline or 2% acetic acid (AA) was slowly infused into the distal colon. Acupuncture treatment was applied 1 hour after the induction of acute visceral hyperalgesia for 15 min. After the application of acupuncture, AWR assessment was performed within 30 min. Then, colon tissue samples were collected 4 hours after instillation of 2% AA after the rats were sacrificed (Figure 1).

### 2.5. Acupuncture Stimulation

The rats in the normal group were not given any other form of treatment after infusion with 1.5 ml of saline but were treated like the animals of the model group. The rats in the model group received the same treatment as those in the ST37 group, without acupuncture treatment after the induction of acute visceral hyperalgesia. The ST37 group was treated with MA at ST37 (5 mm lateral to the anterior tubercle of the tibia and 15 mm below the knee joint) for 15 min like our previous study [29–31], 1 hour after the induction of acute visceral hyperalgesia, by using a small (length: 13 mm, diameter: 0.3 mm) acupuncture needle (Suzhou Hua Tuo Medical Instrument Co., Suzhou, China). Needles were inserted at a depth of 5 mm into the acupoint, and twirling manipulation was performed at 5 min intervals for 30 s. Each needle was bidirectionally rotated 180° at a speed of 2 Hz. The LI11 group received the same treatment at the LI11 point that was located at a depression anterior to the lateral aspect of the elbow. In the ST37 + IGF-1 group, the PI3K agonist IGF-1 (4119-1000, Biovision, 0.5 mg/kg per rat, dissolved in saline) was intraperitoneally injected into the rats 30 min before acupuncture at the ST37 acupoint, and the remaining manipulations were the same as those in the ST37 group. In the IGF-1 group, rats were treated in the same way as those of the ST37 + IGF-1 group but were not treated with acupuncture.

### 2.6. AWR Score

To assess hyperalgesic response, AWR observations were performed within 30 min after the end of acupuncture treatment. Stimulation for colorectal distention (CRD) was conducting while monitoring AWR as previously described [32]. Under light anesthesia induced using anhydrous ether (using 2-3 cotton balls dipped in anhydrous ether placed in a transparent box), a 6 cm distention balloon (constructed using a 6 cm long condom inflated with air) was inserted into the colon. To prevent the balloon catheter from sliding out, it was fixed to the tail with tape. The animal was put in a 20 × 5 × 8 cm acrylic cage and permitted to regain consciousness and acclimatize to the environment for 30 min. To gradually induce four different levels of constant pressure (20, 40, 60, and 80 mmHg), the CRD balloon catheter was connected to a portable sphygmomanometer. CRD was performed for each rat three times at 5 min intervals, with all measurements performed for 20 s at the indicated pressures. AWR scores were recorded in accordance with published scoring criteria [32]: 0, no behavioral response to CRD; 1, immobile during CRD; 2, a mild abdominal muscle contraction, but no lifting of the abdomen; 3, a strong abdominal muscle contraction and lifting of the abdomen, but no lifting of the pelvic structure; and 4, body arching and lifting of the pelvic structure.

The rats were sacrificed at predetermined sampling time, and 1 cm of colon tissue samples at 6 cm from the anal margin was collected 4 hours after instillation of 2% AA. All operations were performed on ice, and the 1 cm colon tissues were divided into three sections and removed quickly into cryopreservation tubes and stored in liquid nitrogen until use for ELISA, western blot, and quantitative real-time PCR.

### 2.7. Inflammatory Cytokine Assessment by ELISA

The levels of tumor necrosis factor (TNF)-*α*, interleukin (IL)-1*β*, and interleukin (IL)-6 in colon tissue were measured using commercially available rat ELISA kits according to the manufacturers' instruction, after the colon tissue was homogenized, and the supernatant was taken. Standard or sample solution (100 *μ*L) was applied to the 96-well polystyrene microplates and incubated for 90 min at 37°C. Then, 10 *μ*L biotinylated antibodies was applied to the wells and incubated for 60 minutes at 37°C. The mixture was then aspirated in each well, and each well was washed with 1 × wash buffer three times. Next, 100 *μ*L of tetramethylbenzidine (TMB) substrate was added to each well and incubated for 10 minutes. 100 *μ*L of stop solution was applied to stop the reaction, and the wells were read at 450 nm.

### 2.8. Quantitative Real-Time PCR

We used an RNA extraction kit (Invitrogen, USA) to extract complete RNA. A High Capacity cDNA Reverse Transcription Kit (TaKaRa, Japan) was used to synthesize cDNA. The procedure for reverse transcription was as follows: 42°C fo 900 s and 98°C for 15 s. Amplification of multiple samples was conducted using SYBR Green (TaKaRa, Japan). Each reaction mixture (20 *μ*L) contained 4 *μ*L of forward primer, 4 *μ*L of reverse primer, 2 *μ*L of cDNA, and 10 *μ*L of Mix SYBR Green. The PCR protocol using the ABI StepOnePlus RT-PCR instrument (Applied Biosystems, USA) was as follows: 40 cycles of 95°C for 30 s, 95°C for 5 s, and 60°C for 30 s, with GAPDH as the internal control [30]. The primers for NGF, TrkA, PI3K, and TRPV1 mRNA detection were predesigned (GenScript, China) as follows: NGF F: 5ʹ- ACT GGA CTA AAC TTC AGC ATT CC-3ʹ, R: 5ʹ-GGG CAG CTA TTG GTT CAG CA-3ʹ; TrkA F: 5ʹ-GCC TAA CCA TCG TGA AGA GTG-3ʹ, R: 5ʹ-CCA AAG CAT TGG AGG AGA GAT-3ʹ; PI3K F: 5ʹ-CCC ACT TCT ATA GCC AAC AAC-3ʹ, R: 5ʹ-GAT ATC TCC CCA GTA CCA TT-3ʹ; Akt F: 5ʹ-CAC AGG TCG CTA CTA TGC CAT GAA G-3ʹ, R: 5ʹ- GCA GGA CAC GGT TCT CAG TAA GC-3ʹ; TRPV1, F: 5ʹ-CCC GGA AGA CAG ACA GCC TGA-3ʹ, R 5ʹ-TTC AAT GGC AAT GTG CAG TGC TG-3ʹ; and GAPDH F: 5ʹ-AGA TGG TGA AGG TCG GTG TGA-3ʹ, R: 5ʹ-CTG GAA GAT GGT GAT GGG TTT CC-3ʹ. Data were processed using the 2^−ΔΔCt^ method.

### 2.9. Western Blotting Analysis

The levels of NGF, TrkA, PI3K, p-Akt/Akt, and TRPV1 in the colon tissues of the rats were detected using western blotting assay. The colon samples were homogenized in protein lysis buffer (RIPA), and equal amounts of protein (50 *μ*g) were electrophoretically resolved on a sodium dodecyl sulfate-polyacrylamide gel (8% separation gel and 5% concentration gel). The resolved proteins were transferred onto a PVDF membrane, and immunoblotting was performed with the following antibodies: NGF (1 : 1000, ab6199, Abcam), TrkA (1 : 1000, ab76291, Abcam), PI3K (1 : 1000, ab151549, Abcam), Akt (1 : 1000, 10176-2-AP, Proteintech), p-Akt (Ser473) (1 : 2000, 66444-1-Ig, Proteintech), and TPRV1 (1 : 500, ab6166, Abcam). The secondary antibodies used were goat anti-mouse IgG (1 : 5000, SA00001-1, Proteintech) and goat anti-rabbit IgG (1 : 5000, HA1001, Huabio), and *β*-actin was used as an internal control (1 : 2500, ab8227, Abcam).

### 2.10. Data Analysis

The results of each study were represented as the mean ± SD. Multiple-group studies were analyzed with one-way analysis of variance, followed by the Tukey honestly significant difference (HSD) post hoc test. *P* < 0.05 was considered statistically significant.

## 3. Results

### 3.1. Effect on AWR Scores

The AWR scores in response to CRD at pressures of 20, 40, 60, and 80 mmHg were recorded and were significantly higher in animals with acute visceral hyperalgesia than in those of the normal control group. After MA treatment at ST37, the AWR scores in the ST37 group were significantly lower than those in the model group (*P* < 0.05). But MA at the LI11 point showed no significant effects compared to the model group (*P* > 0.05), and significant differences were observed between the LI11 and ST37 group (*P* < 0.05). Moreover, the effects of MA at ST37 were inhibited by the administration of the PI3K agonist IGF-1; the ST37 + IGF-1 group showed significant differences when compared to the ST37 group (*P* < 0.05), but not the IGF-1 group (*P* > 0.05; Figure 2).

### 3.2. Downregulation of TNF-*α*, IL-1*β*, and IL-6 after MA at ST37

TNF-*α*, IL-1*β*, and IL-6 expressions were significantly higher in the colons of rats with acute visceral hyperalgesia than in those of healthy rats (*P* < 0.05). MA treatment at ST37, but not LI11, could reduce TNF-*α*, IL-1*β*, and IL-6 expressions (Figure 3).

### 3.3. MA Treatment at ST37 Reduced TRPV1 mRNA Levels in the Colon via PI3K Pathway Induced by NGF

NGF, TrkA, PI3K, and TRPV1 mRNA expressions in the colon of rats with acute visceral hyperalgesia were significantly higher than those in the normal control group. MA treatment at ST37, but not at LI11, could reduce NGF, TrkA, PI3K, Akt, and TRPV1 mRNA expression. Downregulation of PI3K, Akt, and TRPV1 mRNA expression due to MA treatment in the ST37 + IGF-1 group was blocked by IGF-1 treatment; significant differences in PI3K, Akt, and TRPV1 mRNA expression were observed between the ST37 + IGF-1 and ST37 (*P* < 0.05) groups. PI3K, Akt, and TRPV1 mRNA expressions were upregulated by the PI3K agonist IGF-1 in the IGF-1 group, compared to those in the model group (*P* < 0.05). Downregulation of NGF and TrkA mRNA expression by MA treatment at ST37 was still observed, with significant differences between the ST37 + IGF-1 and model groups (*P* < 0.05). NGF and TrkA mRNA expressions in the ST37 + IGF-1 group were not affected by IGF-1 treatment, while there are no differences in NGF and TrkA mRNA expressions between the IGF-1 and model groups (*P* > 0.05; Figure 4).

### 3.4. MA Treatment at ST37 Reduced TRPV1 Protein Expression in the Colon via NGF-Mediated PI3K Pathway Modulation

The expression of NGF, TrkA, PI3K, p-Akt, and TRPV1 proteins was significantly higher in the colons of rats with acute visceral hyperalgesia than in those of healthy controls (*P* < 0.05). MA treatment at ST37, but not LI11, could reduce NGF, TrkA, PI3K, p-Akt, and TRPV1 protein expression. The downregulation of PI3K and TRPV1 protein expressions after MA treatment in the ST37 + IGF-1 group was reversed by treatment with IGF-1. Significant differences in PI3K, p-Akt, and TRPV1 protein expression were observed between the ST37 + IGF-1 and ST37 groups (*P* < 0.05), and no differences were observed between the ST37 + IGF-1 and model groups (*P* > 0.05). PI3K, p-Akt, and TRPV1 protein expression in the IGF-1 group increased significantly after treatment with the PI3K agonist IGF-1, compared to that in the model group (*P* < 0.05). However, downregulation of NGF and TrkA protein expressions due to MA treatment at ST37 was still observed, with significant differences between the ST37 + IGF-1 and model groups (*P* < 0.05). NGF and TrkA protein expressions were not affected by IGF-1 treatment, and there were no significant differences in NGF and TrkA expressions between the IGF-1 and model groups (*P* > 0.05) (Figure 5).

## 4. Discussion

Acupuncture is widely used to alleviate visceral pain in China, owing to its ability to provide pain relief with few side effects such as addictiveness [33, 34]. Several clinical studies have demonstrated the efficacy of acupuncture-moxibustion in visceral pain treatment [10]. MA is commonly used by traditional acupuncturists, and insertion of penetrating needles into acupoints as well as manual rotation of acupuncture needles could enhance its clinical benefits [35–37]. With the increased use of acupuncture in pain control, the mechanism underlying its effects has attracted much attention.

Qi et al. [7, 26] established an acute visceral hyperalgesia model by colorectal instillation with 2% acetic acid, which is a reliable animal model to study the mechanism underlying the effects of acupuncture in the treatment of acute visceral hyperalgesia. In this study, we demonstrated that the AWR scores at a constant pressure of 20, 40, 60, and 80 mmHg of balloon colonic stimulation were higher in the visceral hyperalgesia model group than in the normal group (Figure 2), confirming that the established model of acute visceral hyperalgesia was suitable for subsequent experiments.

Stimulation at specific somatic tissues (acupoints) can long distantly modulate internal organ physiology, and the somatotopy dependent feature of EA in the anti-inflammatory experiment has been reported recently [38]. ST37 is one of the most effective acupoints for treating intestinal diseases including IBS [12, 13], functional constipation [14], intestinal dysfunction [15], and inflammatory bowel disease [16, 17]. EA at ST37 and Zusanli (ST36) could significantly decrease the abnormal increase in AWR scores and magnitude of electromyograms (EMGs) recorded from the rectus abdominis in response to CRD stimulation at 20, 40, 60, and 80 mmHg in chronic visceral hypersensitivity [24, 25] and acute visceral hyperalgesia [7, 26]. The LI11 is also a common acupoint in the clinical treatment of abdominal pain as the *He-*Sea point of the large intestine meridian of hand-Yangming, and acupuncture at LI11 as well as ST37 or some other acupoints could effectively improve functional constipation [14, 18, 39]. However, acupuncture at LI11 showed no obvious effects on proximal colonic movement [40], and its effect was weaker than that of acupuncture at ST37 in the treatment of ulcerative colitis [20] or zymosan-induced colorectal hypersensitivity [19]. In this study, we found similar results. MA at ST37 decreased AWR scores, but LI11 had no significant effect in the treatment of acute visceral hyperalgesia (Figure 2). The analgesic effect of ST37 is better than LI11 and may be associated with the different nerve segments of them. The colonic nerve segment is located at the level of T_6_-L_3_, ST 37 at the level of L_4_-S_2_ [41] and LI11 containing afferents from C_5_ spinal dorsal horn [42]. The nerve segments of colon and ST 37 are relatively near, while LI11 is not. Therefore, MA at ST 37 gets a better analgesic effect than LI11.

The anti-inflammatory effects of acupuncture were a result of a decrease in proinflammatory cytokines (TNF-*α*, IL-1*β*, and IL-6), and improved macroscopic inflammation [43–46]. In this study, MA treatment at ST37 could reduce the expression of TNF-*α*, IL-1*β*, and IL-6, which were upregulated in the colon of rats with acute visceral hyperalgesia (Figure 3). Peripheral injury or inflammation induced the secretion of large amounts of inflammatory mediators, and the expression of IL-1, IL-6, TNF-*α*, and prostaglandin E_2_ (PGE_2_) was significantly elevated in the acute inflammatory visceral pain induced by acetic acid in rats, which contributed to the sensitization of peripheral receptors involved in pain transmission as the levels of TRPV1 and calcitonin gene-related peptide (CGRP) increased [21].

TRPV1 is expressed in extrinsic primary afferents in response to stimulants such as capsaicin, mustard oil, and heat [23]. It is also highly expressed in the bowels and serves as a key regulator of visceral hyperalgesia [10, 27, 47–49]. We previously showed that stimulating at ST37 can enhance jejunal motility in rats and mice [50] and that TRPV1 is partially involved in the acupuncture-mediated modulation of gastric motility [48, 51]. However, the role of TRPV1 in MA analgesia in cases of acute visceral hyperalgesia is unclear. In this study, we found that TRPV1 protein and mRNA expression in rats with acute visceral hyperalgesia were higher than the normal and decreased after MA, which indicated that acupuncture could alleviate visceral pain by mediating the regulation of TRPV1, as observed previously [10, 27].

TRPV1 activity could be regulated by NGF [52, 53]. As a receptor tyrosine kinase, the NGF high-affinity receptor, TrkA, traditionally signals via activation of phospholipase C (PLC*γ*), p42/p44 mitogen-activated protein kinase (ERK), or PI3K [53]. The PI3K/Akt pathway, and not the PLC pathway, is a major pathway downstream of NGF that can participate in sensory hypersensitivity in various animal models [53–56]. Following treatment with acute NGF or peripheral capsaicin injection, TRPV1 activity is mediated via the PI3K/Akt pathway [53, 57]. Akt activity (phosphorylation) is increased in colonic afferent cells in a colitis state and is coexpressed with TRPV1 and TrkA [58]. Thus, the NGF-PI3K-TRPV1 axis likely plays a prominent role in colonic hyperalgesia. Previous study found that activating the PI3K/Akt pathway by enhancing the expression of p-Akt (Ser473) can exert anti-inflammatory effects [59], and EA can affect the PI3K/Akt signaling pathway by regulating the p-Akt level and the ratio of p-Akt/Akt [60]. A recent study found that stimulating at ST36 could trigger mast cell activity, activate the NGF/TrkA/TRPV1 peripheral afferent pathway, and alleviate visceral hypersensitivity in chemical inflammatory model rats [61]. But it is still unknown whether acupuncture mediates the expression of TRPV1 through the pathway downstream of NGF/TrkA. In the present study, MA at ST37 could substantially reduce the levels of NGF, TrkA, PI3K, p-Akt, and TRPV1, while the LI11 acupoint treatment could not (Figures 4 and 5). The effect of MA at ST37 is better than LI11; maybe the reason is that the spinal ganglion segment of ST37 is adjacent to colorectum, while LI11 is not [19].

IGF-1, as a PI3K agonist, is frequently used to verify the mechanism of the PI3K/Akt pathway [62–64]. The biological function of IGF-I is mainly mediated by IGF-I receptor. The activation of the IGF-I receptor by its endogenous agonist causes receptor autophosphorylation and activation of intrinsic tyrosine kinase, which subsequently phosphorylates a host of intracellular substrates including insulin-receptor substrate-1 (IRS-1). Phosphorylation of IRS-1 leads to stimulation of PI3K and the activation of serine/threonine kinase Akt [65]. And we found that MA at ST37 could reduce the levels of PI3K, p-Akt, and TRPV1. The effect was blocked by treating with the PI3K agonist IGF-1before MA, PI3K p-Akt, and TRPV1 protein expression increased significantly (Figure 5). The effects of MA treatment at ST37 on AWR scores were reduced by IGF-1 treatment before MA (Figure 2), which indicated that acupuncture could alleviate acute visceral hyperalgesia in rats by depressing TRPV1 expression via the NGF-induced PI3K/Akt pathway.

## 5. Limitation

Our present findings have provided evidence that MA analgesia to acute visceral hyperalgesia is related to acupoint specificity, for MA at ST37 ameliorates behavioral hyperalgesia by TRPV1 via the NGF-induced PI3K/Akt pathway in rats with acute visceral hyperalgesia, while MA at LI11 shows no effect. But there are some limitations of the current study. The dose-effect of the analgesic effect of these two acupoints for visceral pain is unknown. And it is still not known how acupuncture signals are transmitted and cause changes in the PI3K/Akt pathway of target organs to achieve analgesic effect. TRPV1 is regulated by many factors, and its potential mechanism for alleviating inflammatory pain is complex [66–68]. In order to further confirm the role of TRPV1 in the MA analgesia, more family members of the PI3K/Akt pathway and other TRPV1 activating substances should be explored, while the pathogenesis of acute visceral hyperalgesia is complex and varying.

## 6. Conclusion

MA at ST37, but not at LI11, could significantly decrease the AWR scores in rats with acute visceral hyperalgesia. Our results indicate that the mechanism underlying the analgesic effects of acupuncture at ST37 on acute visceral hyperalgesia likely involves a reduction in TRPV1 expression, which is regulated by the PI3K/Akt pathway, induced by NGF. This may help understand the mechanism of acupuncture in the treatment of acute visceral pain.

## Figures and Tables

**Figure 1:** Acupuncture treatment and experimental procedure. (a) Location of the LI11 acupoint (LI11, or Quchi; black arrow, upper image) and the ST37 acupoint (ST37, or Shangjuxu; black arrow, lower image). (b) Experimental schedule. Rats in the LI11 and ST37 groups received manual acupuncture for 15 minutes; normal control rats were restrained manually for the same duration. Rats in ST37+IGF-1 group were intraperitoneally injected IGF-1 30 min before manual acupuncture.

**Figure 2:** AWR scores after MA at ST37 in rats with acute visceral hyperalgesia. AWR scores in response to CRD with colon balloon stimulation pressures of (a) 20, (b) 40, (c) 60, and (d) 80 mmHg were tested. Data are expressed as the mean ± SD (*n* = 6 for each group. ^*∗*^*P* < 0.05 vs. model group; ^&^*P* < 0.05 vs. ST37 group).

**Figure 3:** Effect of MA at ST37 on proinflammatory cytokine expression. The levels of (a) TNF-*α*, (b) IL-1*β*, and (c) IL-6 in rat colon tissues. Data are expressed as the mean ± SD (*n* = 6 for each group. ^*∗*^*P* < 0.05 vs. model group; ^&^*P* < 0.05 vs. ST37 group); IL-1*β*, interleukin-1*β*; IL-6, interleukin-6; TNF-*α*, tumor necrosis factor-*α*.

**Figure 4:** Effects of MA stimulation on NGF, TrkA, PI3K, Akt, and TRPV1 mRNA expressions in the colon of rats with acute visceral hyperalgesia. Data are expressed as the mean ± SD (*n* = 3 for each group. ^*∗*^*P* < 0.05 vs. model group; ^&^*P* < 0.05 vs. ST37 group; ^#^*P* < 0.05 vs. ST37 + IGF-1 group).

**Figure 5:** Effects of MA stimulation on NGF, TrkA, PI3K, TRPV1, and p-Akt protein expressions in the colons of rats with acute visceral hyperalgesia. Representative blots for NGF, TrkA, PI3K, TRPV1, p-Akt, and densitometry analyses were performed (a–e). To confirm equal sample loading, *β*-actin was used for normalization (the level of the p-Akt was counted by the ratio of p-Akt/Akt). Data are expressed as the mean ± SD (*n* = 6 for each group. ^*∗*^*P* < 0.05 vs. model group; ^&^*P* < 0.05 vs. ST37 group; ^#^*P* < 0.05 vs. ST37 + IGF-1 group).

## Data Availability

The data used to support the findings of this study are included within the article.

## Supplementary Materials

Supplementary Materials The article was reported by following the guidelines of “The ARRIVE Guidelines for Reporting Animal Research [69]” and the ARRIVE guidelines checklist was supplied in the supplementary file.
